RETRACTED

# Double‐blind, randomized, placebo‐controlled pilot study of the phosphodiesterase‐3 inhibitor cilostazol as an adjunctive to antidepressants in patients with major depressive disorder

**DOI:** 10.1111/cns.13731

**Published:** 2021-09-21

**Authors:** Mahmoud S. Abdallah, Ahmed N. Ramadan, Hend Omara‐Reda, Noha O. Mansour, Mohamed A. Elsokary, Hozaifa K. Elsawah, Shimaa Abdelsattar Zaki, Hend E. Abo Mansour, Esraa M. Mosalam

**Affiliations:** ^1^ Department of Clinical Pharmacy Faculty of Pharmacy University of Sadat City Sadat City Egypt; ^2^ Department of Neuropsychiatry Faculty of Medicine Menoufia University Shebin El‐Kom Egypt; ^3^ Clinical Pharmacy and Pharmacy Practice Department Faculty of Pharmacy Mansoura University Mansoura Egypt; ^4^ Department of Biostatistics High Institute of Public Health Alexandria University Alexandria Egypt; ^5^ Department of Clinical Biochemistry and Molecular Diagnostics National Liver Institute Menoufia University Shebin El‐Kom Egypt; ^6^ Department of Biochemistry Faculty of Pharmacy Menoufia University Shebin El‐Kom Egypt

**Keywords:** adjunctive therapy, cilostazol, CREB/BDNF, inflammatory markers, major depressive disorder

## Abstract

**Aims:**

Cilostazol (CLS) has shown antidepressant effect in cardiovascular patients, post‐stroke depression, and animal models through its neurotrophic and antiinflammatory activities. Consequently, we aimed to investigate its safety and efficacy in patients with MDD by conducting double‐blind, randomized, placebo‐controlled pilot study.

**Methods:**

80 participants with MDD (DSM‐IV criteria) and Hamilton Depression Rating Scale (HDRS) score >20 were treated with CLS 50 mg or placebo twice daily plus escitalopram (ESC) 20 mg once daily for six weeks. Patients were evaluated by HDRS scores (weeks 0, 2, 4, and 6). Serum levels of CREB1, BDNF, 5‐HT, TNF–α, NF‐ κB, and FAM19A5 were assessed pre‐ and post‐treatment.

**Results:**

Co‐administration of CLS had markedly decreased HDRS score at all‐time points compared to the placebo group (*p* < 0.001). Early improvement, response, and remission rates after 6 weeks were significantly higher in the CLS group (90%, 90%, 80%, respectively) than in the placebo group (25%, 65%, 50% respectively) (*p* < 0.001). Moreover, the CLS group was superior to the placebo group in modulation of the measured neurotrophic and inflammatory biomarkers.

**Conclusion:**

CLS is safe and effective short‐term adjunctive therapy in patients with MDD with no other comorbid conditions.

Trial registration ID:NCT04069819.

## Graphical abstract

Cilostazol treatment improve the expression of neurotrophic factors and decreases the expression of inflammatory cytokines. The neurotrophic and anti‐inflammatory properties of cilostazol responsible for its antidepressant action. Cilostazol is a safe and effective short‐term adjunctive therapy in patients with major depressive disorder with no other comorbid conditions.

RETRACTED

## 1 INTRODUCTION

Major depressive disorder (MDD) is a common mental disorder with serious socioeconomic consequences on daily life and health care costs.^1^ Although the advent of newer monoamine pathways targeted antidepressants, nearly fifty percent of patients have no response to the first‐line antidepressant therapy.^2^ Therefore, augmentation strategy using agents with novel mechanism of action and therapeutic targets at the start of the therapy could provide additional therapeutic benefits for patients with MDD.^3^

Several studies have shown the importance of cyclic adenosine monophosphate (cAMP) cascade in MDD.^4^ It has been noted that the cAMP is downregulated in MDD and upregulated by antidepressant.^5^ Medications that increase the expression level of cAMP could activate the transcription of cAMP response element‐binding protein (CREB).^6^ As a result, activation of CREB increases the expression of brain‐derived neurotrophic factor (BDNF), which has an important function in neuronal development and synaptic plasticity.^7^, ^8^ Several findings have demonstrated that BDNF may be involved in the antidepressants therapeutic action.^9^, ^10^

On the other hand, cumulative evidence has shown that an increased inflammatory response of the central nervous system (CNS) plays a critical role in MDD pathophysiology.^11^, ^12^ Pro‐inflammatory cytokines such as interleukin‐1beta (IL‐1β), IL‐6, and tumor necrosis factor‐α (TNF‐α) are elevated in patients with MDD and decreased after therapy.^11^, ^12^, ^13^, ^14^ Furthermore, these cytokines can disrupt the synthesis of 5‐hydroxytryptamin (5‐HT)^15^ and glutamatergic transmission, which are profoundly implicated in the pathophysiology MDD.^16^ FAM19A5 is a novel peptide‐like chemokine that is highly expressed in the brain and developed during neurogenesis.^17^ Increased serum level of FAM19A5 has been linked to neuroinflammation and neurodegeneration in patients with MDD.^18^

Cilostazol (CLS), a selective phosphodiesterase‐3 (PDE‐3) inhibitor, acts as an antiplatelet agent with neurotrophic and anti‐inflammatory properties.^19^, ^20^ It has strong pleiotropic effects by restoring cAMP/CREB signaling and stimulating BDNF gene expression.^21^, ^22^ It showed antidepressant action in post‐stroke depression and in animal models through inhibition of neurodegeneration and promotion of neurogenesis.^22^, ^23^ Besides CLS can overcome the inflammation‐based hypothesis for the development of MDD by its ability to suppress TNF‐mediated nuclear factor kappa B (NF‐κB) and the release of cytokines.^20^, ^24^ These findings suggest it to be beneficial adjunctive therapy for patients with MDD.

RETRACTED

In this trial, we supposed that CLS could exert antidepressant effect in patients with MDD. Therefore, we aimed to investigate its safety and efficacy in the treatment of patients with MDD with no other comorbid conditions by conducting double‐blind, randomized, placebo‐controlled pilot study of CLS as adjunctive agent. Furthermore, we aimed to evaluate its neurotrophic and antiinflammatory activities in those patients.

## 2 MATERIALS AND METHODS

### 2.1 Study design

This was a single center, prospective, double‐blinded, randomized, placebo‐controlled pilot study, which was conducted over six weeks to compare CLS with placebo, adjunctive to escitalopram (ESC) in patients with MDD.

### 2.2 Participants

From August 2019 to April 2021, patients aged 20–60 years for both genders were recruited from Menoufia University Hospital, Egypt. Diagnosis was confirmed according the Diagnostic and Statistical Manual of Mental Disorders‐IV (DSM–IV) based on MINI Neuropsychiatric Interview.^25^, ^26^ Patients with Hamilton Depression Rating Scale (HDRS) score >20 were eligible.^27^ Patients’ medical history was recorded to guarantee the absence of drugs and diseases that could interact or interfere with the study. The study was registered on ClinicalTrials.gov (NCT04069819) and approved by the ethics committee of the Faculty of Medicine, Menoufia University (NEUR22021). The patients and their representatives signed a written informed consent in an agreement with the measures stated by the local ethical committee. The study was conducted in compliance with Helsinki Declaration.

Patients have physical illness that could interfere with the study, drug allergy or contraindications, bipolar I or II disorders, personality disorder, anxiety disorder, eating disorder, substance abuse, receiving electroconvulsive therapy, taking other psychotropic drugs except ESC in the past month, serious suicide risk, psychotic symptoms, pregnant females, and breastfeeding mothers have been excluded. Routine blood, hematochemical, and urine analyses were conducted at baseline to exclude physical illness like anemia, thyroid dysfunction, diabetes, renal, hepatic or heart diseases, and neoplasm.

### 2.3 Sample size

This study was designed as a pilot, proof‐of‐concept study. Sample size calculation was based on Teare et al. who recommended the sample size of a pilot trial to be 70 measured subjects (35 per group) in order to reduce the imprecision around the estimate of the standard deviation.^28^ Considering a 10% attrition rate, sample size of 40 subjects in each group was calculated.

RETRACTED

### 2.4 Randomization and blinding

The randomization code generation was done by randomization block method using SPSS software by an independent party (allocation ratio 1:1) to receive either CLS or placebo plus ESC. Allocation Concealment was done using sequentially numbered enclosed opaque packets. Placebo tablets were supplied by Sigma Pharmaceutical Company, Menoufia, Egypt, and they were indistinguishable from CLS in their size, color, and shape. The patients, the physician who referred the patient, care provider, the statistician, and the assessor were all blinded to treatment allocation. Patients were excluded from the trial if they missed their trial medication for a week.

### 2.5 Intervention

Patients were randomly assigned to receive either CLS 50 mg tablet twice daily or placebo tablets in the same way adjunctive to ESC 20 mg once daily for six consecutive weeks. The medications were distributed by the pharmacy, and the returned pills were counted.

### 2.6 Outcomes

The primary outcome was the 17‐items HDRS score was recorded at the baseline and after 2, 4, and 6 weeks from the starting the medications. Early improvement was defined as 20% reduction in HDRS total score in the first 2 weeks, response rate (≥50% decrease in the HDRS total score), and remission rate (HDRS total score ≤7). Moreover, a checklist was used to monitor the adverse drug reactions and medication adherence. The patients were followed up weekly by phone to assess their compliance with the medications in addition to counting the remaining pills. The secondary outcome measurements were the serum levels of CREB1, BDNF, 5‐HT (5‐hydroxytryptamine), TNF‐α, NF‐ κB, and FAM19A5 that measured pre‐and post‐treatment to assess the biological effect of the used drugs.

### 2.7 Measurements

Morning blood samples (5 ml) were drawn from all patients by venepuncture in plain vacutainers at the same time (8:00 a.m.) following an eight‐hour fast. The vacutainers were then centrifuged at 4500×*g* for 15 min to obtain separated serum samples, which were transferred to Eppendorf tubes and maintained in a deep freezer at −80℃ until analysis. Serum levels of CREB1, BDNF, 5‐HT, TNF–α, NF‐ κB, and FAM19A5 were measured using specific commercial ELISA kits purchased from MyBioSource, Inc. (USA). The measurements were carried out according to the manufacturers’ instructions using Biotek ELx800 UV‐Vis Microplate Reader (USA).

### 2.8 Statistical analysis

IBM^®^ SPSS^®^ Statistics version 22 software (IBM Corp., Armonk, NY, USA) was used to analyze the data. Continuous variables were expressed as mean ± standard deviation (SD), and categorical variables were expressed as number (percentage). For continuous variables, the Student's t test was used for independent samples, and if the *t*‐tests’ normality assumptions are not met, the Wilcoxon rank sum test was used. The Shapiro‐Wilk and Kolmogorov‐Smirnov tests were used to assess the assumption of normality. For categorical data, the chi‐square test or Fisher's exact test was used as appropriate. Treatment efficacy tests were done at two‐sided significance level of 0.05. Mixed‐effects model repeated measures (MMRM) analysis of covariance (ANCOVA) was used for comparing the end‐point score in HDRS total score. The change between the two groups in HDRS score was compared using two‐way analysis of variance (ANOVA) with‐repeated measures (group as inter‐subject factor) with four measurements as within‐subject factor. Bonferroni correction was done for multiple comparisons. Moreover, ANCOVA was done to compare the change in the biomarkers after six weeks in the two groups. Graphs were performed using GraphPad Prism 6.01 software (GraphPad Software, La Jolla CA, USA).

RETRACTED

## 3 RESULTS

Figure 1 shows that after screening 140 patients for selection criteria, 60 patients were excluded from the study because they had another active medical problem or refused to participate in the study. Eighty eligible patients were assigned to either CLS plus ESC (*n* = 40) or placebo plus ESC (*n* = 40). Table 1 shows the demographic and baseline data of the patients. Two weeks after the beginning of the study, eight patients dropped out due to non‐compliance with the procedures; four were in the placebo group and four were in the CLS group. These dropped subjects were included in the HDRS analysis but were omitted from the biomarker analysis. The HDRS baseline scores between the two groups were not statistically different (mean ± SD for placebo was 22.6 ± 2.6, for CLS was 22.9 ± 2.3, *t* = 0.289, df = 78, *p* = 0.387).

**FIGURE 1:** Flow diagram of study participants

**TABLE 1:** Demographic and baseline characteristics of the participants

	Placebo group (*n* = 40)	Cilostazol group (*n* = 40)	Statistical value
Age (years)	38.1 ± 10.02	37.05 ± 9.4	*t* = 0.456, df = 78, *p* = 0.324
Gender			
Male	9 (22.5%)	10 (25%)	X^2^ = 0.209, df = 1, *p* = 0.647
Female	31 (77.5%)	30 (75%)	X^2^ = 0.209, df = 1, *p* = 0.647
Smoking	12 (30%)	10 (25%)	X^2^ = 0.044, df = 1, *p* = 0.833
Weight (kg)	76.93 ± 8.67	77.88 ± 8.56	*t* = 0.567, df = 78, *p* = 0.286
Height (cm)	173.38 ± 10.96	172.68 ± 10.84	*t* = 0.433, df = 78, *p* = 0.333
BMI (kg/m^2^)	23.74 ± 1.67	23.18 ± 1.57	*t* = 1.12, df = 78, *p* = 0.133
Marital status			
Single	15 (37.5%)	13 (32.5%)	X^2^ = 0.334, df = 1, *p* = 0.563
Married	15 (37.5%)	18 (45%)	X^2^ = 0.334, df = 1, *p* = 0.563
Divorced	10 (25%)	11 (27.5%)	X^2^ = 0.334, df = 1, *p* = 0.563
HDRS score	22.6 ± 2.6	22.9 ± 2.3	*t* = 0.289, df = 78, *p* = 0.387
Prothrombin time (second)	12 ± 0.7	11 ± 0.87	*t* = 0.239, df = 78, *p* = 0.406
Episodes of depression			
First	30 (75%)	31 (77.5%)	X^2^ = 0.209, df = 1, *p* = 0.647
Second	10 (25%)	9 (22.5%)	X^2^ = 0.209, df = 1, *p* = 0.647
Drugs used in last episode			
Paroxetine	3 (7.5%)	1 (2.5%)	X^2^ = 0.201, df = 1, *p* = 0.653
Fluoxetine	3 (7.5%)	1 (2.5%)	X^2^ = 0.201, df = 1, *p* = 0.643
Escitalopram	4 (10%)	4 (10%)	X^2^ = 0.201, df = 1, *p* = 0.653

Notes

Data presented as mean ± SD. Chi‐square test was used for categorical data and student *t*‐test was used for continuous data.

RETRACTED

Abbreviations: BMI, body mass index; HDRS score, Hamilton Depression Rating Scale score.

### 3.1 Effect on HDRS Score (primary outcome)

The MMRM analysis showed a statistically significant decrease in the HDRS total score in CLS group compared to the placebo group after 2, 4, and 6 weeks of the treatment ((least squares mean difference [LSMD] – 2.83, *p* = 0.001), [LSMD] – 3.74, *p* = 0.001), ([LSMD] – 3.99, *p* = 0.001), respectively) as shown in Figure 2. The two‐factor ANOVA analysis showed that the difference between the two treatments was statistically significant, as indicated by the effect of group; the inter‐subject factor (F(1, 70) = 60.67, *p* = 0.02, η_2_ = 0.64). The difference between the two treatments was significant as indicated by the effect of groups‐by‐time interaction (F(3, 210) = 56.89, *p* = 0.000, η_2_ = 0.448). The early improvement was a statistically significant higher in the CLS group than the placebo group (90% in the CLS group *vs* 25% in the placebo group, *p* < 0.001). The CLS group also showed statistically significant improved response to the treatment by the fourth and sixth week. The response rate for CLS group was 90% *vs* 65% for placebo group after six weeks (*p* <0.001); number need to treat (NNT) = 4. Remission rate was 80% for CLS group vs 50% for placebo group after six weeks (*p* < 0.001; NNT = 3.33) as shown in Table 2.

**FIGURE 2:** Baseline‐to‐Endpoint Changes in Hamilton Depression Rating Scale (HDRS) Total Score. Data presented as mean ± SD. Mixed‐effects model repeated measures (MMRM) analysis of covariance (ANCOVA) was used for comparing the end‐point score in HDRS total score. HDRS, Hamilton Depression Rating Scale (HDRS)

**TABLE 2:** Comparison of outcome measures between the two groups

Outcome	Placebo group (*n* = 40)	Cilostazol group (*n* = 40)	*p*‐Value of Fisher's exact test	Risk ratio (95% CI)
Number (%) of early improvers	10 (25%)	36 (90%)	<0.001	0.286 (0.140–0.582)
Number (%) of responders at week 4	20 (50%)	32 (80%)	<0.001	0.456 (0.206–1.07)
Number (%) of responders at week 6	26 (65%)	36 (90%)	<0.001	0.123 (0.018–0.824)
Number (%) of remitters	20 (50%)	32 (80%)	<0.001	0.345 (0.124–0.96)

Notes

Early improvement: at least 20% decrease in Hamilton depression rating scale (HDRS) score by week 2. Response: at least 50% decrease in HDRS score. Remission: HDRS score of ≤7. Fisher's exact test was used for comparison of proportions.

RETRACTED

### 3.2 Effect on neurotrophic and inflammatory biomarkers (secondary outcome)

The difference between the CLS and the placebo groups, in the baseline serum levels of CREB1, BDNF, 5‐HT, TNF–α, NF‐ κB, and FAM19A5, was statistically nonsignificant (Table 3). Using ANCOVA after six weeks of treatment, the CLS group showed a statistically substantial increase in the serum levels of CREB1, BDNF, and 5‐ HT compared with the placebo group ((F (1, 70) = 79.43, *p* = 0.001, η_2_ = 0.531), (F (1, 70) =69.3, *p* = 0.004, η_2_ = 0.497), and (F (1, 70) =67.3, *p* = 0.001, η_2_ = 0.49), respectively). On the other hand, the serum levels of TNF–α, NF‐ κB, and FAM19A5 were statistically significant lower in the CLS group compared to the placebo group ((F (1, 70) = 118.19, *p* = 0.002, η_2_ = 0.629), (F (1, 70) = 108.86, *p* = 0.003, η_2_ = 0.608), and (F (1, 70) = 99.34, *p* = 0.001, η_2_ = 0.586), respectively).

**TABLE 3:** Baseline‐to‐endpoint changes in selected neurotrophic and inflammatory biomarkers in the two groups

Groups	Placebo group (*n* = 36)			Cilostazol group (*n* = 36)			*P* value Week 6*
Parameters	Baseline	Week 6	*P* value**	Baseline	Week 6	*P* value**	
CREB1 (ng/ml)	1.82 ± 0.6	3.88 ± 1.2	*p* = 0.002	1.74 ± 0.57	6.13 ± 1.97	*p* = *0.002*	*p* = 0.001
BDNF (ng/ml)	10.7 ± 3.26	25.9 ± 8.24	*p* = 0.002	11.67 ± 3.62	39.66 ± 12.3	*p* = 0.002	*p* = 0.004
5‐HT (ng/ml)	60.23 ± 18.02	110.26 ± 35.91	*p* = 0.001	63.18 ± 20.05	134.94 ± 40.9	*p* = 0.001	*p* = 0.001
TNF‐α (pg/ml)	11.12 ± 3.42	7.16 ± 2.19	*p* = 0.001	11.58 ± 3.58	4.45 ± 1.44	*p* = 0.001	*p* = 0.002
NF‐ κB (ng/ml)	3.12 ± 0.99	1.56 ± 0.5	*p* = 0.001	3.18 ± 1.01	0.65 ± 0.21	*p* = 0.001	*p* = 0.003
FAM19A5 (ng/ml)	2.995 ± 0.95	1.27 ± 0.40	*p* = 0.001	2.93 ± 0.98	0.79 ± 0.22	*p* = 0.001	*p* = 0.001

Notes

Data presented as mean ± SD. Student *t*‐test was used for dependent variables and analysis of covariance (ANCOVA) was used to compare the change after six weeks in the two groups.

Abbreviations: CREB1: cAMP response element‐binding protein, BDNF: brain derived neurotrophic factor, 5‐HT: 5‐hydroxytryptamine, TNF‐α: tumor necrosis factor alpha, NF‐ κB: nuclear factor kappa B, FAM19A5: Chemokine‐like protein.

RETRACTED

*Between groups comparison after 6 weeks.

**Within group comparison.

After six weeks of treatment, CREB1, BDNF, and 5‐HT serum levels were statistically significant higher in comparison with their baseline data as reflected by the effect of groups‐time interaction ((F (1, 70) = 49.45, *p* = 0.002, η_2_ = 0.414), (F (1, 70) = 66.67, *p* = 0.002 η_2_ = 0.488), and (F (1, 70) = 55.75, *p* = 0.001, η_2_ = 0.443), respectively). In contrary, the serum levels of TNF–α, NF‐ κB, and FAM19A5 were statistically significant lower compared with their baseline data as indicated by the effect of groups‐time interaction ((F (1, 70) = 55.67, *p* = 0.001, η_2_ = 0.442), (F (1, 70) = 65.67, *p* = 0.001, η_2_ = 0.484), and (F (1, 70) = 70.45, *p* = 0.001, η_2_ = 0.501), respectively).

### 3.3 Clinical side effects

The difference between the CLS and the placebo groups in terms of the frequency of the side effects was statistically nonsignificant (Table 4). Over the period of the trial, 15 side effects were recorded; the most common of which was headache (20% placebo, 22.5% CLS). The other reported side effects were transient and spontaneously resolved.

**TABLE 4:** Frequency of side effects in the study groups

Side effects	Placebo group *N* (%)	Cilostazol group *N* (%)	*P value*
Decreased appetite	4 (10%)	5 (12.5%)	*p* = 0.78
Increased appetite	4 (10%)	3 (7.5%)	*p* = 0.78
Fatigue	3 (7.5%)	2 (5%)	*p* = 0.78
Dry mouth	3 (7.5%)	3 (7.5%)	*p* = 1.00
Headache	8 (20%)	9 (22.5%)	*p* = 0.78
Tremors	1 (2.5%)	2 (5%)	*p* = 0.78
Dizziness	4 (10%)	5 (12.5%)	*p* = 0.78
Insomnia	6 (15%)	7 (17.5%)	*p* = 0.78
Runny nose	2 (5%)	4 (10%)	*p* = 0.6
Muscle aches	3 (7.5%)	6 (15%)	*p* = 0.42
Nausea	3 (7.5%)	5 (12.5%)	*p* = 0.78
Abdominal pain	4 (10%)	6 (15%)	*p* = 0.692
Heartburn	3 (7.5%)	6 (15%)	*p* = 0.42
Diarrhea	4 (10%)	5 (12.5%)	*p* = 0.78
Sexual dysfunction	8 (20%)	5 (12.5%)	*p* = 0.42

Note

Fisher's exact test was used for comparison of proportions.

## 4 DISCUSSION

The previously published human studies regarding the antidepressant effect of CLS have been involved patients with cardiovascular diseases associated with MDD or post‐stroke depression.^29^, ^30^ Therefore, and to our knowledge, this study is the first double‐blind, randomized, and placebo‐controlled pilot trial that evaluates the adjunctive role of CLS in the management of patients with MDD with no other comorbid conditions.

It has been reported that using combined medications at the beginning of the treatment of MDD patients may provide additional therapeutic benefits as ~50% of the patients do not respond to the first‐line antidepressants.^2^, ^3^ Although study designs make direct comparison a difficult issue, the response rate of 90% in the CLS combination group is consistent to that of previous studies (89%–92%) including simvastatin,^31^ metformin,^32^ or pentoxifylline^12^ as adjuvant therapies in MDD patients over 6 and 12 weeks. Furthermore, the remission rate of 80% in our study is also consistent with the 59%–85% remission rates in the above‐mentioned trials.^12^, ^31^, ^32^ Moreover, the rapid reduction in the HDRS score in the first two weeks in the CLS group is in consistent with previous studies, which reported that adjuvant PDE inhibitors and anti‐inflammatory agents could lead to a rapid‐onset antidepressant effect in MDD patients.^12^, ^31^, ^33^ Regarding the response and remission rates in the placebo group, which were 65% and 50%, they were also comparable to the previously reported response and remission rates for monotherapy in two published studies, which were 58%–76%, and 27%–64%, respectively.^12^, ^34^, ^35^

Several evidences indicated a correlation between MDD and both PDEs and inflammatory pathways.^11^, ^36^ Thus, higher response and remission rates in the CLS combination group could be related to its neurotrophic and antiinflammatory actions, which resulted in a significant increase in the CREB1, BDNF, and 5‐HT serum levels along with a significant decrease in the TNF‐α, NF‐κB, and FAM19A5 serum levels.^20^, ^22^, ^29^, ^37^, ^38^ CLS could improve brain plasticity by modulating the levels of neurotrophic factor, like BDNF, via CREB activation as reported in preclinical and clinical studies.^22^, ^29^, ^39^ Different clinical studies have showed that BDNF could mediate the antidepressants’ therapeutic activities by enhancing the neuronal plasticity as MDD patients have a decreased level of BDNF, which was restored to the normal levels by the antidepressant therapy.^9^, ^10^

The high serum level of FAM19A5 in MDD has been reported, which reflects the activation of neuroinflammatory processes and increased production of pro‐inflammatory cytokines such as TNF‐α, IL‐6, or IL‐1β.^18^, ^40^ Moreover, preclinical studies have shown that theses cytokines could activate the N‐methyl‐D‐aspartate receptor (NMDA) receptors, thus increasing excitotoxicity and reducing neurogenesis as well as the BDNF.^41^, ^42^ Our findings were in agreement with other studies, which have shown that CLS directly inhibits cytokines’ expression triggered by NF‐κB activation.^24^, ^38^, ^43^ As a consequence, the reduced level of the pro‐inflammatory cytokines resulted in an increased bioavailability of 5‐HT through regulation of its metabolic pathways.^44^, ^45^

Furthermore, ESC monotherapy could increase the levels of CERB/BDNF as reported in preclinical and clinical studies.^46^, ^47^, ^48^ ESC also has antiinflammatory effect, which mediated by reducing the pro‐inflammatory cytokines.^49^ These changes were reflected in a high response rate to ESC, which is consistent with previous studies indicated that ESC was effective in reducing depressive symptoms when compared to placebo.^50^, ^51^

The improved antidepressant effect in the combination group could be attributed to the addition of CLS. Therefore, our study suggests CLS as an effective and safe adjunct to ESC in patients with MDD and provided considerable proof for its efficacy in patients with MDD without other comorbid conditions. This notion was particularly reinforced by previous study, which recommended CLS as an alternative to milnacipran for the treatment of patients with post‐stroke depression as it led to a decrease in HDRS after switching from milnacipran to CLS (100 mg/day).^29^ In addition, CLS has been reported to have potential efficacy in geriatric MDD patients with cerebrovascular problems.^52^ These outcomes suggested CLS as a preferred drug for treatment of mild to moderate depression in cardiovascular patients who undergoing angioplasty and requiring adjuvant antiplatelet therapy.^30^ In addition, it is consistent with the results of preclinical studies, which indicate that CLS produced antidepressant‐like activities when given either alone or in combination with other psychotropic agents.^23^, ^39^

Despite the promising results regarding the use of CLS in the management of MDD, it is still early to be considered as a primary treatment for MDD due to some study limitations including the short follow‐up period and the small sample size. Moreover, measurement of corticosterone level is recommended to evaluate the alteration of hypothalamic‐pituitary‐gonadal (HPA)‐axis dysregulation as both neuroinflammation and neurotrophic activities are directly mediated by HPA‐axis. Therefore, more comprehensive, larger scale, multicenter, and longer duration clinical studies are required to confirm the efficacy of CLS in the treatment of MDD.

RETRACTED

## 5 CONCLUSION

Co‐administration of CLS, a selective phosphodiesterase‐3 inhibitor, with ESC to patients with MDD enhanced the antidepressant therapeutic effects through its neurotrophic and anti‐inflammatory properties. This was reflected clinically by early improvement, better response, and higher remission rate. In addition, the detection of biological markers including CREB/BDNF and FAM19A5 may be clinically useful for the assessment of antidepressant response. Theses outcomes suggest CLS to be promising adjunctive candidate to antidepressants, but further investigations with larger sample size and longer follow‐up durations are recommended to overcome the limitations of this study.

## CONFLICT OF INTEREST

The authors have no conflicts of interest to declare.

## Data Availability

The data that support the findings of this study are available on request from the corresponding author. The data are not publicly available due to privacy or ethical restrictions.
